# Development of a Sensitive Quality Evaluation System for Chinese Outstanding Female Boxers

**DOI:** 10.1155/2022/4664938

**Published:** 2022-07-30

**Authors:** Haibo Zhong, Xiangui Bu

**Affiliations:** School of Competitive Sports, Shandong Sport University, Rizhao 276800, China

## Abstract

**Objective:**

To construct an evaluation system for the sensitivity quality of outstanding Chinese female boxers and to develop comprehensive evaluation criteria for the sensitivity quality of outstanding female boxers.

**Methods:**

Using literature method, Telfer method, expert interview method, and experimental test method to analyze the special sensitivity quality structural elements of female boxers.

**Results:**

The evaluation indexes of female boxers' sensitivity quality consisted of three structural elements: ability to change movements, ability to change direction, and balance ability; the evaluation index system of female boxers' sensitivity quality, including 3 primary indexes and 11 measurement indexes, in which the weights of the primary indexes of female boxers' special sensitivity quality were 0.44 for the ability to change movements (0.22 for 1 min dodge defense, 0.22 for 1 min combination punching sandbag 0.21, 30 s standing push-up 0.21, and 30 s leg change jumping punch 0.19), the ability to change direction 0.39 (30 s continuous head hold squat 0.16, 1 min 3 m sides slide touch 0.29, 20 s repeated side slide 0.28, 10 m *∗* 4 round trip run 0.24, and 1 min quadrant jump 0.19), and balance ability 0.17 (15 s rotating and then walking forward 5 m 0.51, carrying legs to support balance 0.49), the ability to change movements has the largest proportion in the sensitivity quality of female boxers, followed by the ability to change direction and balance ability.

**Conclusion:**

Based on the constructed evaluation index system, 11 individual indexes' evaluation criteria and four levels of comprehensive evaluation criteria for the sensitivity quality of female boxers were established by using the deviation method and percentile method.

## 1. Introduction

In the 32nd Tokyo Olympic Games, Chinese female boxers won two silver medals, but there is still a big gap compared with traditional boxing powerhouses such as Cuba and Russia, and this competition also revealed many problems, such as lack of variation in fighting style, poor rhythm, and lack of flexibility in footwork. Boxing has high requirements for agility, especially the ability to move with footwork [1, 2], and as a skill-driven combat sport, the environment in which boxing players are involved is constantly changing, requiring them to make decisions and counterattacks according to their opponents' technical and tactical actions [3–5], which puts higher requirements on the agility of female boxers. The literature review found that there is a lack of research on the evaluation of the sensitivity quality of female boxers, so it is necessary to conduct an in-depth exploration of the sensitivity quality of boxers. The construction of an evaluation system for the sensitivity quality of excellent female boxers can effectively evaluate the development level of sensitivity quality of female boxers and provide a theoretical basis for the targeted improvement of sensitivity quality training of female boxers.

## 2. Research Objectives and Methods

### 2.1. Research Subjects

In this study, the sensitivity quality of female boxers from Shandong Province boxing team and Shandong Sports College was used as the study object. 34 athletes were selected as the sample (Table1), with the age range (19.2 ± 1.66 years) and the training time (5.69 ± 1.57 years).

### 2.2. Research Methods

#### 2.2.1. Literature Method

Various domestic and foreign materials on the development of boxing, training of boxing programs, sports measurement, and evaluation with sports were obtained through the library of Shandong Institute of Physical Education and Sports, Super Star Library, etc.; several databases such as China Knowledge Network, Baidu Academic, Google Academic, Pubmed, Web of Science were used to obtain relevant literature at home and abroad. To obtain policy documents about boxing through the official websites of boxing at home and abroad, we used “agility”, “boxing agility”, “combat sports agility”, “boxing training”, etc., for searching. The Chinese keywords searched included “agility”, “boxing”, “boxing athlete selection”, “boxing agility”, and “boxing training”, etc.

#### 2.2.2. Expert Interview Method

After determining the topic and concept of the thesis, interviews were conducted with experts in boxing coaching and teaching by means of telephone consultation, WeChat, and on-site interviews, etc. In order to ensure the smooth development of the study, experts in the following two areas were selected: regarding the selection of topics, test items and methods for the evaluation criteria of boxers' sensitive quality structure, two senior coaches of boxing training, and five experts in physical education, experts in teaching and other fields, were interviewed; three boxing coaches and 10 outstanding boxing athletes were interviewed about the training of boxing athletes and the implementation of the evaluation test index in practice. Through the summary of the opinions of experts from various aspects, the structure system of sensitivity quality was initially constructed.

#### 2.2.3. Telfer Method

Combined with the initial sensitivity quality indexes established by expert interviews, the Telfer method was used to issue questionnaires to experts of boxing programs, and after the investigation of the two questionnaires, the sensitivity quality indexes of female boxers were initially determined.

#### 2.2.4. Experimental Test Method

Through the screening of boxing sensitivity quality indexes by experts, the test indexes that can determine the athletes' sensitivity were initially determined, and then the athletes who participated in the test were tested on the initial indexes.

## 3. Results and Analysis

### 3.1. Preliminary Establishment of a Structural Model for the Evaluation of Sensitivity Quality of Female Boxers

Combined with the characteristics of boxing sports, a preliminary index system of sensitivity quality of female boxers was established. The boxing-specific sensitivity quality indexes with high correlation and significant influence were screened out, and the preliminary indexes of boxing-specific sensitivity quality included three primary indexes of changing action ability, changing direction ability and balance ability, and 20 secondary indexes (Table 2).

### 3.2. Expert Findings and Analysis

The experts interviewed were involved in various fields such as boxing sports training, physical training, physical fitness measurement and evaluation, and biomechanics research, which could be done to minimize the influence of subjective tendencies and one-sidedness. The recall rate was 81% for the first round and 100% for the second round, both of which met the needs of the study [6].

#### 3.2.1. Modification of the First Round of Questionnaire Indicators

Twenty items were initially selected as test indexes for the special sensitivity quality of female boxers, and the degree of influence of each index on the sensitivity quality of boxers was divided into five levels: very important, important, average, unimportant, and very unimportant, and the first round of expert questionnaires was designed. Based on the experts' scores of each index, 18 indexes with scores higher than 3.75 were initially selected [7], as shown in Table 3 (1 means selected, 0 means discarded by you). The second round of expert questionnaires was finally designed by combining the experts' suggestions.

#### 3.2.2. Modification of Indicators in the Second Round of Questionnaire

The first round of experts' judgment on the importance of each index, combined with experts' opinions, was summarized and analyzed to reformulate the boxers' special sensitivity quality expert questionnaire, and the second round of opinion solicitation was conducted on the selected indexes; the results are shown in Table 4; all indexes were basically approved by experts, and no new modification suggestions were made.

#### 3.2.3. Preliminary Establishment of Special Sensitivity Quality Index Structure of Female Boxers

Through summarizing two rounds of expert opinions, screening and modifying part of the preliminary indexes, and optimizing and organizing the unscientific indexes, and based on the analysis of the authority coefficient, coordination degree, and positive coefficient of expert opinions, a special sensitivity quality evaluation structure including 13 test indexes and three elements was initially determined, and the three elements are the elements of changing movement ability, changing direction ability, and balance ability.

### 3.3. The Establishment of Special Sensitivity Quality Test Index System for Female Boxers

Boxing special sensitivity quality test indexes should not only reflect the requirements of boxing for special sensitivity quality, but also make the test indexes accurately reflect the reality of boxing sports, so as to achieve less but more precise result. Therefore, it is necessary to further screen the initially determined test indexes and select the ones with strong operability and simplicity. In order to determine the final measurement indexes, principal component analysis was applied, and a bivariate correlation test was done before factor analysis, and from Table 5, it can be seen that the KMO value was 0.74, and the value of the correlation test between variables was moderate in size, which was more suitable for factor analysis [8].

#### 3.3.1. Factor Loadings Statistics

Exploratory factor analysis was done on the initially selected 13 indicators, and three main components were obtained when the selected eigenvalues were greater than 1. The 1 min jump back drill gear indicator had high loadings in both the first and second factors, spanning two factors, and the reliability of the test results was relatively low due to the difference in difficulty caused by the difference in height of the athletes during the test, so the indicator was considered for deletion. Then, the second exploratory factor analysis was done for the remaining 12 indicators, and it was concluded that the loadings of 1 min double swing jump rope in the second factor were lower than 0.6, so it was deleted [8], and then the third exploratory factor analysis was conducted to obtain Table 6, from which we can see that the loadings of 11 indicators were above 0.6, among which the loadings of 1 min quadrant jump in the first and second factors exceeded 0.5, but the loading value in the second factor reached 0.6 or more, and combined with the expert's suggestion, this indicator can be classified as the second factor, and all the remaining indicators can be retained.

#### 3.3.2. Factor Analysis of Different Special Sensitivity Qualities

Selecting the number of indicators with eigenvalues greater than 1, the three principal components obtained and the cumulative contribution rate reached 74.923%; these factors can summarize 74.923% of the overall information. It is reasonable to consider these three factors as the main constituents of the special sensitivity quality of female boxers (Table 7).

The three initial factors obtained were orthogonally rotated to make them more consistent with the actual meaning, and the indicators with higher factor loadings were obtained on each principal component. The factor attribution of individual indicators was determined based on the absolute value of the loadings of each tested indicator, and the experts' opinions were combined to name the special sensitivity factors for female boxers (see Table 8).

### 3.4. Establishment of Evaluation Index System

The contribution rate of the variance of each component is generally expressed as the percentage of variance of the initial eigenvalue, and the more important the component is, the larger its corresponding contribution rate is. Therefore, the weights of each principal component can be replaced by the contribution rate of the variance. The weight coefficients of the primary and secondary indicators of female boxers were calculated based on the contribution of each factor in the total explained variance of each tested indicator and the matrix value of the principal component score coefficients.

As can be seen from Table 9, the weight coefficients of the first level indicators are arranged in the order from largest to smallest: the element of ability to change movements (0.44), the element of ability to change direction (0.39), and the element of balance ability (0.17). It can be seen that the index of ability to change movements quickly has the largest weight coefficient in the sensitivity quality of female boxers, followed by the ability to change directions quickly, and the balance ability is smaller, but it is also the main factor that constitutes the sensitivity quality of female boxers.

#### 3.4.1. The Establishment of Special Sensitivity Quality Evaluation Criteria for Female Boxers

*(1) Development of Individual Index Standards*. In order to scientifically and accurately judge the development degree and level of each single index of female boxers, so as to make a comprehensive and integrated evaluation of the athletes' sensitivity, it is necessary to develop the evaluation criteria of each test index. The indicators are quantified in order to discover individual differences in athletes' sensitivity quality. In this study, the “standardized percentage method” was used to evaluate the individual indicators, and an evaluation table was designed for each indicator. In order to facilitate the comparison among the indicators, the measured values were first standardized by using the *T* standard score method, where ±3 standard deviations were selected to cover 99.73% of the total rating range, calculated as follows:

(1) $$\begin{array}{c} T=50\pm \frac{100\left(X-\bar{X}\right)}{6S}, \end{array}$$

where *x* is the measured data, *T* is the standard percentage, and *S* is the standard deviation of each test item as well as the mean, and the score standard of each individual index is calculated.

As can be seen from Table 10, the larger the *T* value, the higher the level of each index of female boxers and the higher the level of their special sensitivity qualities.

*(2) Development of Comprehensive Index Criteria*. In order to accurately evaluate the special sensitivity of female boxers, this study used the principal component analysis to determine the weights of primary and secondary indicators and used the weighted summation method to evaluate the individual indicators and the comprehensive sensitivity quality indicators, assuming that the ability of female boxers in all aspects is the dependent variable (Y), and derived the evaluation model of each dimension of sensitivity quality and overall.

Model for each dimension:

(2) $$\begin{array}{c} Y_{\text{Ability to switch movements}}=0.221\times 4+0.213\times 11+0.209\times 3+0.195\times 2+0.162\times 8,\\ Y_{\text{Change of direction capability}}=0.287\times 5+0.281\times 10+0.239\times 7+0.193\times 6,\\ Y_{\text{Balancing ability}}=0.506\times 1+0.494\times 9. \end{array}$$

The comprehensive evaluation model is

(3) $$\begin{array}{c} Y_{\text{Overview}}=0.44\;Y_{\text{Ability to switch movements}}+0.39\;Y_{\text{Change of direction capability}}+0.17\;Y_{\text{Balancing ability}}\text{.} \end{array}$$

According to the measurement and evaluation theory, the percentile method and the deviation method are two more common methods of rating evaluation, and this study uses the percentile method, which is calculated by the following formula:

(4) $$\begin{array}{c} P_{i}=X_{i}\frac{j}{S_{i}}\left(\frac{i\cdot N}{100}-B_{i}\right), \end{array}$$

where the *i*th percentile is denoted by *P*_*i*_, *S*_*i*_ is the frequency of the group in which *P*_*i*_ is located, *X*_*i*_ denotes the minimum of the median value of the *i*th percentile group, *B*_*i*_ denotes the frequency of the previous group of *X*_*i*_, *j* is the group distance, and the sample size is denoted by *N*.

The SPSS22.0 statistical program was used to calculate the corresponding scores of P15, P65, and P90, and each grade interval was divided for each index of sensitivity quality and comprehensive quality score. Finally, a comprehensive evaluation table of the sensitivity quality of female boxers was determined (see Table 11).

#### 3.4.2. Application of Evaluation Criteria

Taking female boxer Jing X as an example, the raw scores corresponding to the 11 indexes measured by the original scores of 5 m walking forward after rotation, standing props, continuous dodging defense, 1 min 3 m sliding touch line on both sides, 1 min quadrant jump, 10 m *∗* 4 round trip run, 30 s continuous head squat, closed-eye leg carry support, repeated side sliding, and 1 min combination punching sandbag were 34.57, 27.31, 43.42, 43.34, 43.46, 42.35, 33.71, 33.71, 60.19, 40.08, and 21.65, respectively. By substituting the scores of these 11 indexes into the evaluation model of the influence factors of the agility quality and the comprehensive model, the athlete's agility quality and comprehensive agility quality scores were calculated, and the scores of change of movement, change of direction, and balance ability were 14.5, 14.6, 14.7, 14.8, and 14.9, respectively. Referring to Table 11, we found that the athlete's agility quality was within the range of passing grade, and the development of all aspects of agility quality was balanced but not high. Therefore, it is necessary to strengthen the special practice of sensitivity quality in normal training, so as to improve the overall level of sensitivity quality.

### 3.5. Analysis and Discussion

#### 3.5.1. Ability to Change Movements

If boxers want to take the initiative on the field, they must have good punching speed and be able to take the initiative to hit the opponent to score, and they need to have a high level of physical fitness [9], and if boxers want to complete various technical movements with high quality, such as stomp and turn power, body twisting power, and continuous power striking, strength quality is an important guarantee [9, 10], and this kind of integration of the external manifestation of the fusion of “power” and “speed” is the athlete's fast movement speed. Fast and heavy punches often give the opponent a heavy blow, so that the opponent loses combat power, which is conducive to control the pace of the game; boxers in various confrontations need to continue to improve their ability to quickly complete a variety of technical actions to gain the advantage of time, using the time difference to seize the first opportunity.

#### 3.5.2. Ability to Change Direction

The new rule changes make the “fast” element of winning more critical. Fast boxing can destroy the opponent's center of gravity, and fast and flexible movement of footwork is an effective way to surprise, interfere, and create opportunities to win the game initiative. During the game, fast movement is the core of the game, which can effectively control the distance between attack and defense and the pace of the game.

#### 3.5.3. Balancing Ability

The element of balance is an important part of the overall agility quality, although it has a small proportion in the overall agility quality. In competition, boxers have to maintain the ability to maintain the space and position in which the body is positioned, and the athletes have to maintain control of themselves under the conditions of various changing movements. For example, when attacking, the body loses its center of gravity when punching empty and needs to adjust its body balance in time and maintain a stable center of gravity during physical confrontation, and when attacking or defending, boxers need to quickly adjust their dynamic balance when moving quickly in order to complete various subsequent movements. In particular, athletes need to have a strong ability to maintain body balance after being hit by heavy punches.

## 4. Conclusions and Recommendations

1. The structural model of the evaluation indexes for the sensitivity quality of female boxers was determined. This study established a theoretical structural model of the specific agility quality evaluation index system for female boxers and concluded that the agility quality evaluation indexes consist of three structural elements: ability to change movements, ability to change direction, and balance ability.
2. The evaluation index system of female boxers' agility quality was created. The evaluation index system of female boxers' agility quality was determined under the guidance of evaluation principles, including 3 primary indexes and 11 measurement indexes, in which the weights of the primary indexes of female boxers' special agility quality were 0.44 for the ability to change movements (0.22 for 1-minute dodge defense, 0.21 for 1-minute combination punching sandbag, 0.21 for 30 s standing push-up, and 0.19 for 30 s leg change jumping out of punch), (30s leg change jumping punch 0.19), ability to change direction 0.39 (30s continuous head hold squats 0.16, 1 min 3 m sides slide touch 0.29, 20 s repeated side slide 0.28, 10 m *∗* 4 round trip run 0.24, and 1 min quadrant jump 0.19) and balance ability 0.17 (15 s rotate and then walk forward 5 m 0.51, carry leg support balance 0.49), ability to change movements. The ability to switch movements accounted for the largest proportion of the agility quality of female boxers, followed by the ability to change direction and balance ability.
3. The evaluation criteria of female boxers' agility quality were developed. Based on the constructed evaluation index system, 11 individual indexes' evaluation criteria and four levels of comprehensive evaluation criteria of female boxers' agility quality were established by using the deviation method and the percentile method, and the evaluation model was validated, and the results showed that the established criteria could be used for the assessment of female boxers' agility quality.

## Figures and Tables

**Table 1:** Number of athletes in each level.

Level	National grade II	National level	Fitness level
Number of people	17 people	12 people	5 people
Total	34 people		

**Table 2:** Preliminary selection of sensitive quality evaluation index system.

Tier 1 indicators	Tier 2 indicators
A. Ability to changemovements	A1 30 s change legs jumping out of the punch
	A2 1-minute dodge defense
	A3 30 s sit-ups
	A4 1 min jump back drilling gear
	A5 10 s push-ups
	A6 1 min hitting sandbag
	A7 30 s standing push-ups
	A8 30 s continuous head hold squat

B. Ability to changedirection	B1 Illinois run
	B2 1 min 3 m sliding contact line on both sides
	B3 1-minute quadrant jump
	B4 10 m *∗* 4 round trip run
	B5 repeated side slide step
	B6 1 min double swing jump rope

C. Coordination andbalance ability	C1 standing on one foot
	C2 lifting leg support balance
	C3 closed eyes in place
	C4 walking balance beam
	C5 15 s rotate and walk 5 m to the right
	C6 15 s rotate and walk 5 m to the left

**Table 3:** Statistical table of the first round of expert index screening results (*n* = 13).

Specialized sensitive quality indicators	Average value	Standard deviation	Selection status
A change of action ability	4.54	0.52	1
B change of direction capability	4.38	0.51	1
C balancing ability	4.69	0.48	1
A1 30 s change legs jumping out of the punch	4.15	0.69	1
A2 1-minute dodge defense	4.46	0.78	1
A3 30 s sit-ups	3.15	0.69	0
A4 1 min jump back drilling gear	3.92	0.76	1
A5 10 s push-ups	3.43	0.83	0
A6 1 min hitting sandbag	4.00	0.82	1
A7 30 s standing push-ups	3.85	0.69	1
A8 30 s continuous head hold squat	4.46	0.52	1
B1 Illinois run	3.15	0.76	0
B2 1 min 3 m sliding contact line on both sides	3.08	0.49	0
B3 1-minute quadrant jump	4.46	0.52	1
B4 10 m *∗* 4 round trip run	4.23	0.60	1
B5 repeated side slide step	4.31	0.48	1
B6 1 min double swing jump rope	4.15	0.56	1
C1 standing on one foot	3.85	0.56	1
C2 lifting leg support balance	4.46	0.78	1
C3 stepping in place with eyes closed	3.57	0.80	0
C4 walk the balance beam	4.31	0.48	0
C5 15 s rotate and walk 5 m to the right	4.00	0.71	1
C6 15 s rotate and walk 5 m to the left	3.85	0.56	1

**Table 4:** Statistical table of the second round of expert index screening results (*n* = 13).

Test index	Average value	Standard deviation	Coefficient of variation
A change of movement ability	4.62	0.52	0.11
B ability to change direction	4.92	0.28	0.06
C balance ability	4.92	0.28	0.06
A1 30 s leg change jumping punch	4.23	0.6	0.14
A2 1 min dodge defense	4.15	0.38	0.09
A3 1 min combination punching sandbag	4.31	0.48	0.11
A4 30 s standing push-ups	4.77	0.44	0.09
A5 30 s continuous head hold squat	4.31	0.75	0.17
A6 1 min jumping back drill stall	3.87	0.44	0.11
B1 1 min 3 m sliding touch line on both sides	4.31	0.48	0.11
B2 1 min quadrant jump	4.62	0.51	0.11
B3 10 m *∗* 4 round trip run	4.31	0.48	0.11
B4 repeated side slide step	3.85	0.38	0.10
B5 1 min double swing jump rope	4.31	0.48	0.11
C1 balance with leg lift	4.46	0.52	0.12
C2 15 s rotate and walk forward 5 m	4.85	0.38	0.08

**Table 5:** KMO and Bartlett's test table.

KMO sampling suitability quantity		0.74
Bartlett's sphericity test	Approximate cardinality	253.89
	Degree of freedom	55.00
	Significance	0.00

**Table 6:** Factor rotation load matrix.

Indicator name	Ingredients		
	1	2	3
1 min dodge defense	0.885		
1 min combination punching sandbag	0.851		
30 s standing push-ups	0.836		
30 s leg change jumping punch	0.778		
30 s continuous head squat	0.649	0.465	
1 min 3 m or so sliding touch bar		0.962	
20 s repeated side slides		0.944	
10 m *∗* 4 round trip run		−0.803	
1 min quadrant jump	0.515	0.647	
15 s rotate and walk forward 5 m			−0.829
Lift leg support balance			0.809

**Table 7:** Total explained variance of specific sensitivity quality indicators for female boxers.

Ingredients	Initial eigenvalue			Extraction of the sum of squares of loads			Sum of squared rotating loads		
	Total	Percentage of variance	Cumulative (%)	Total	Percentage of variance	Cumulative (%)	Total	Percentage of variance	Cumulative (%)
1	5.097	46.34	46.34	5.097	46.339	46.339	3.61	32.818	32.818
2	1.879	17.08	63.42	1.879	17.079	63.418	3.251	29.556	62.374
3	1.266	11.51	74.92	1.266	11.505	74.923	1.38	12.549	74.923
4	0.669	6.09	81.01						
5	0.599	5.45	86.45						
6	0.454	4.13	90.59						
7	0.442	4.02	94.60						
8	0.307	2.79	97.39						
9	0.145	1.32	98.71						
10	0.1	0.91	99.62						
11	0.042	0.39	100.00						

**Table 8:** Classification and naming of principal components.

Principal components	High load index	Factor naming
1	1 min dodge defense	Changing the action factor
	1 min combination punching sandbag	
	30 s standing push-ups	
	30 s leg change jumping punch	
	30 s continuous head squat	

2	1 min 3 m both sides slide touch line	Change of direction factor
	20 s repeated side slides	
	10 m *∗* 4 round trip run	
	1 min quadrant jump	

3	15 s rotate and walk forward 5 m	Balance factor
	Lift leg support balance	

**Table 9:** Table of special sensitive quality weighting values.

Factor name	Indicators	Weights	
Transformation action factor	1 min dodge defense	0.221	0.44
	1 min combination punching sandbag	0.213	
	30 s standing push-ups	0.209	
	30 s leg change jumping punch	0.195	
	30 s continuous head squat	0.162	

Change direction factor	1 min 3 m both sides slide touch line	0.287	0.39
	20 s repeated side slides	0.281	
	10 m *∗* 4 round trip run	0.239	
	1 min quadrant jump	0.193	

Balance factor	15 s rotate and walk forward 5 m	0.506	0.17
	Lift leg support balance	0.494	

**Table 10:** Single index evaluation table of special sensitivity quality of female boxers.

Score	X1	X2	X3	X4	X5	X6	X7	X8	X9	X10	X11
100	2.26	156.54	26.07	264.37	57.51	57.16	7.91	41.46	21.02	52.14	100.97
95	2.45	152.17	25.18	254.72	56.05	55.24	8.19	40.29	20.24	50.96	97.39
90	2.64	147.80	24.29	245.07	54.59	53.32	8.47	39.13	19.46	49.77	93.82
85	2.83	143.42	23.40	235.42	53.13	51.39	8.74	37.96	18.68	48.59	90.25
80	3.03	139.05	22.51	225.77	51.67	49.47	9.02	36.80	17.90	47.41	86.68
75	3.22	134.68	21.62	216.12	50.21	47.55	9.30	35.63	17.13	46.22	83.11
70	3.41	130.31	20.73	206.46	48.75	45.63	9.58	34.46	16.35	45.04	79.54
65	3.61	125.94	19.84	196.81	47.29	43.71	9.86	33.30	15.57	43.86	75.96
60	3.80	121.57	18.95	187.16	45.83	41.78	10.14	32.13	14.79	42.68	72.39
55	3.99	117.20	18.06	177.51	44.37	39.86	10.41	30.97	14.01	41.49	68.82
50	4.18	112.83	17.17	167.86	42.91	37.94	10.69	29.80	13.23	40.31	65.25
45	4.38	108.46	16.28	158.21	41.45	36.02	10.97	28.63	12.45	39.13	61.68
40	4.57	104.09	15.39	148.56	39.99	34.10	11.25	27.47	11.67	37.94	58.11
35	4.76	99.72	14.50	138.91	38.53	32.17	11.53	26.30	10.89	36.76	54.54
30	4.96	95.35	13.61	129.26	37.07	30.25	11.81	25.14	10.11	35.58	50.96
25	5.15	90.98	12.72	119.61	35.61	28.33	12.08	23.97	9.33	34.40	47.39
20	5.34	86.61	11.83	109.95	34.15	26.41	12.36	22.80	8.56	33.21	43.82
15	5.54	82.24	10.94	100.30	32.69	24.49	12.64	21.64	7.78	32.03	40.25
10	5.73	77.86	10.05	90.65	31.23	22.56	12.92	20.47	7.00	30.85	36.68
5	5.92	73.49	9.16	81.00	29.77	20.64	13.20	19.31	6.22	29.66	33.11

*Note.* X1 = 15 seconds to rotate and then walk forward 5 meters, X2 = 30 seconds to change legs and jump out of the fist, X3 = 30 seconds to stand up, X4 = 1 minute to dodge defense, X5 = 1 minute to slide both sides of 3 meters to touch the line, X6 = 1 minute to quadrant jump, X7 = 10 m *∗* 4 round trip run, X8 = 30 seconds to continuously hold the head squat, X9 = move legs to support balance, X10 = repeat side slide, X11 = 1 minute to combine the fist to hit the sandbag.

**Table 11:** Comprehensive rating scale for special sensitivity qualities of female boxers (weighted).

Indicators	Excellent	Good	Qualified	Difference
Change of movement ability	≥32.19	24.40–32.18	11.54–24.39	＜11.54
Ability to change direction	≥29.06	23.21–39.05	10.42–23.20	＜10.42
Balance ability	≥12.04	9.19–12.03	5.44–9.18	＜5.44
Overall score	≥73.66	56.80–73.65	27.40–56.79	＜27.4
Theoretical percentage	10	25	50	15

## Data Availability

All the data used in this study are to be accessed by request to the corresponding author.

## Additional Points

*Limitations*An index system for evaluating the sensitivity quality of Chinese female boxers was established to make the measurement and evaluation of the sensitivity quality of female boxers more scientific, but the applicability of the evaluation was not determined because the study sample was limited and empirical tests were not conducted with outstanding foreign female boxers.

## References

[1] Kim K. J., Song H. S., Yoon D. H., Fukuda D. H., Kim S. H., Park D. H. (2018). Amateur boxer (%) lactate (%) physical fitness (%) training (%) *β*-alanine. *Journal of Exercise Rehabilitation*.

[2] Sienkiewicz-Dianzenza E., Maszczyk Ł. (2019). The impact of fatigue on agility and responsiveness in boxing. *Biomedical Human Kinetics*.

[3] Davis P., Benson P. R., Pitty J. D., Connorton A. J., Waldock R. (2015). The activity profile of elite male amateur boxing. *International Journal of Sports Physiology and Performance*.

[4] Bruzas V., Kamandulis S., Venckunas T., Snieckus A., Mockus P. (2018). Effects of plyometric exercise training with external weights on punching ability of experienced amateur boxers. *The Journal of Sports Medicine and Physical Fitness*.

[5] Kim K.-J., Song H. S., Min S. K. (2016). Body composition and specific physical fitness profiles of the Korean national amateur boxers. *Exercise Science*.

[6] Wu Z., Wu P., Su Z. (2014). *Modern Social Survey Methods*.

[7] Chen X. (2001). *Principles and Methods of Sport Science Research*.

[8] Wu M. L. (2010). *Operation and Application of Structural Equation Modeling-AMOS*.

[9] Gao G. (2014). *Survey Analysis of the Application of Selection Indexes for Youth Boxers in Liaoning Province*.

[10] Hu Y., Yu L. (2004). Research on the monitoring index of sports quality training of chinese boxing olympic training team members. *Journal of Beijing Sports University*.

